# Posterior Lumbar Plexus Block Anesthesia for Elderly Patients with Lower Limb Fracture

**DOI:** 10.1155/2022/8494796

**Published:** 2022-06-20

**Authors:** Zhenwen Xu, Songpeng Li, Jianhua Wu, Yun Fu

**Affiliations:** ^1^Department of Traditional Chinese Medicine and Traumatology, Huizhou Hospital of Traditional Chinese Medicine, No. 1 Dongsheng Road, Huicheng District, Huizhou, Guangdong, China 516001; ^2^Department of Orthopedics, Huizhou Third People's Hospital, No. 1 Dongsheng Road, Huicheng District, Huizhou, Guangdong, China 516001

## Abstract

The incidence rate of lower limb fractures is high and has increased over the recent years, which affects the physical and mental health and the daily activities of patients. Lower limb fractures are often treated surgically. Therefore, an effective anesthesia regimen is crucial for a smooth and stable operation. To investigate the efficacy of posterior lumbar plexus block anesthesia during surgery for elderly patients with lower extremity fractures. In total, patients were divided into study and control groups. Anesthesia was administered by posterior lumbar plexus nerve block in the study group and epidural anesthesia in the control group. Hemodynamic parameters, anesthesia condition, pain level (VAS), and adverse effects were measured in both groups before anesthesia (T0), at anesthesia induction (T1), 30 min into the operation (T2), and at the end of the operation (T3). At T0, there were no significant differences in MAP and HR between the study and control groups. However, MAP and HR in the study group were significantly lower than those in the control group at T1, T2, and T3. The BIS value of the study group at each time point after anesthesia was significantly lower than that of the control group. The onset and induction time of anesthesia in the study group were also significantly shorter than those in the control group. Preoperative VAS scores did not differ between the study and control groups. However, the VAS scores of the study group at each time point were significantly lower than those of the control group. There was no significant difference in the incidence of adverse reactions between the two groups. Our results suggest that anesthesia with posterior lumbar plexus block surgery for lower extremity fractures in elderly patients can maintain hemodynamic stability and reduce block onset time, anesthesia induction time, and pain.

## 1. Introduction

The incidence of lower limb fractures is high and has increased over the recent years due to the rise in traffic accidents, aerial work, and an aging population, thereby threatening the physical and mental health of patients as well as their ability to perform daily activities [1, 2]. Lower limb fractures are often treated surgically, as it promotes healing and can improve limb function. Therefore, an effective anesthesia regimen is crucial for a smooth and stable operation [3, 4].

At present, the main anesthesia methods for lower extremity fracture surgery are general anesthesia and epidural anesthesia, but there are large hemodynamic fluctuations during the operation. In addition, most elderly patients have other medical conditions, poor health, and tolerance that increase the risk of surgery [5, 6]. Posterior lumbar plexus block anesthesia is increasingly used. This anesthesia method is simple, can minimize the impact on the physiological function of the body, and can avoid large hemodynamic fluctuations. These features are key to ensuring effective and safe surgery [7, 8].

Therefore, this study investigated the effect of posterior lumbar plexus block anesthesia on elderly patients with lower limb fractures through a randomized controlled study.

## 2. Materials and Methods

### 2.1. Patient Selection

Between 1 January 2020 and 31 July 2021, 137 elderly patients with lower limb fractures were enrolled. The eligible patients according to inclusion and exclusion criteria were divided into the study and control group based on a simple random number table. The protocol of current study was approved by the ethic committee of Huizhou Hospital of Traditional Chinese Medicine. All patients signed the informed consent form.

### 2.2. Inclusion Criteria

Patients with lower limb fractures and types identified through CT and other examinations, classified as ASA II or III, aged ≥60 years, and who provided informed consent were included.

### 2.3. Exclusion Criteria

Patients with a pathological fracture; a fracture complicated with other fractures; organic lesions of the kidney, liver, or other organs; mental system lesions or diseases; and an allergic constitution or history of allergies to the study drugs were excluded.

### 2.4. Anesthesia Methods

After entering the room, the venous channel was quickly opened to assist the patient into the lateral decubitus position. A posterior lumbar plexus nerve block anesthesia was administered in the study group. The nerve stimulator was set at a 1 Hz frequency and 1 mA current. The positive electrode was placed under the connecting puncture needle, and the negative electrode was placed under the anterior superior iliac spine. The line was drawn parallel to the spine through the posterior superior iliac spine as the connecting line of the iliac spine. The intersection point of the two lines was the puncture point. The nerve puncture needle was inserted perpendicularly into the skin at the puncture point, and the current was adjusted to a threshold of 0.3 mA after inducing a contraction of the quadriceps femoris. The puncture was successful after confirming no contractile activity of the quadriceps muscle, and then, the puncture needle was fixed. After blood and other liquids were no longer pumping back out, the local anesthetic was injected, and 20 mL of 1% lidocaine (Xi'an Fenghua Pharmaceutical Co. Ltd., SFDA ZhunZi H61020861) +30 mL of 0.5% ropivacaine (Ruiyang Pharmaceutical Co., Ltd., SFDA ZhunZi H20183151) was injected to assist the patient into a supine position.

Epidural anesthesia was administered in the control group, and the epidural puncture was performed through the space between L1 and L2 using a No. 18 puncture needle. If there was a sense of frustration, an epidural catheter was inserted. First, 3 mL of 2% lidocaine was administered, and then, 10 mL of 0.75% ropivacaine was injected. The blocking plane was viewed 15 min later. If the blocking plane was lower than T11, another 5 mL of 0.75% ropivacaine was administered.

### 2.5. Observation Indicators

Hemodynamic indices (e.g., heart rate (HR) and mean arterial pressure (MAP)) before anesthesia (T0), during anesthesia induction (T1), 30 min into the operation (T2), and at the end of the operation (T3) were measured in both groups using a Philips INTELLIVUE multifunctional monitor. The anesthetic conditions were also recorded, including the bispectral index (BIS) at 5, 15, and 30 min of anesthesia, the block onset time, and the anesthesia induction time. BIS values ranged from 0 to 100, with a lower score indicating deeper inhibition of the cerebral cortex. Pain severity (VAS) was measured before the operation, immediately after the operation, and 6, 24, and 48 h after the operation. The VAS scores ranged from 0 to 10, with a higher score indicating more pain. Finally, adverse reaction incidences were recorded.

### 2.6. Statistical Analysis

Data were analyzed by SPSS 22.0 (IBM Corp., Armonk, NY, USA), including quantitative data (mean ± standard deviation), *t*-test, and enumeration data (*n* (%)), *χ*^2^ test. The two-sided *P* values < 0.05 indicated statistical significance.

## 3. Results

### 3.1. Baseline Data

In this study, 25 patients were excluded due to less than 60-year-old. A total of 112 patients were divided into two groups, each group contained 56 patients. The study group contained 29 men and 27 women, and the average age was 73.97 ± 12.04 (range, 61–87) years. Based on the American Society of Anesthesiologists (ASA) classification, 30 cases were class II, and 26 were class III. The average body mass index (BMI) was 22.06 ± 3.96 (range, 17.4–26.6) kg/m^2^. There were 19 tibiofibular fracture cases, 18 femoral shaft fracture cases, 16 femoral neck fracture cases, and 3 cases classified as “other.”

The control group had 31 men and 25 women, and the average age was 75.06 ± 10.87 (range, 60–89) years. There were 32 ASA class II cases and 24 class III cases. The average BMI was 21.99 ± 4.11 (range, 6.9–27.2) kg/m^2^. There were 16 tibiofibular fracture cases, 21 femoral shaft fracture cases, 14 femoral neck fracture cases, and 5 cases classified as “other.” Clinical data, such as sex, age, the ASA classification, BMI, and the fracture type, were balanced and comparable between the groups (*P* > 0.05).

### 3.2. Hemodynamic Index Levels

At T0, MAP and HR did not differ between the study and control groups (*P* > 0.05). However, at T1, T2, and T3, MAP and HR were significantly lower in the study group than those in the control group (*P* < 0.05; Table 1).

### 3.3. Anesthesia Measurements

The BIS values in the study group were lower than the control group at all time points after anesthesia administration. The anesthesia onset and induction times were also significantly shorter in the study group than those in the control group (*P* < 0.05; Table 2).

### 3.4. VAS Scores

The VAS score before surgery did not differ between the study and control groups. However, the VAS scores of the study group at all time points were significantly lower than those in the control group (*P* < 0.05; Table 3).

### 3.5. Adverse Reactions

The adverse reaction incidence rate did not differ between the two groups (*P* > 0.05; Table 4).

## 4. Discussion

The incidence of lower extremity fractures is high, and surgery is the mainstay of treatment. However, it can cause hemodynamic fluctuations during surgery, resulting in increased blood pressure and increased heart rate, thereby increasing the risk of surgery in the elderly [9, 10], and the anesthesia scheme can directly affect the safety of the surgery and postoperative limb function rehabilitation [11]. Therefore, the optimal anesthesia protocol for lower limb fracture surgeries remains an important topic.

Epidural anesthesia is commonly used in lower extremity fracture surgery, but there are still large hemodynamic fluctuations during the operation, which limits its wide clinical application [12]. New research has indicated that the lumbar plexus mainly includes the anterior branch of the 12^th^ thoracic nerve and the anterior branches of the 1^st^–4^th^ lumbar nerves. Further, the nerve branches are mostly distributed in the muscles and skin of the medial side of the foot, leg, and thigh (i.e., the quadratus lumborum and iliopsoas muscles) [13, 14]. A lumbar plexus block includes the anterior and posterior lumbar plexus blocks and has broad use. However, the anterior lumbar plexus block is only suitable for patients undergoing lower extremity surgery with or without a tourniquet for a short time [15, 16]. In this study, posterior lumbar plexus block anesthesia was used in elderly patients with lower extremity fractures. The results showed that patients who received posterior lumbar plexus block had significantly lower BIS values than those who received epidural anesthesia. Compared with epidural, patients who received posterior lumbar plexus block also had shorter block onset time and anesthesia induction time, indicating that posterior lumbar plexus block was effective and shortened anesthesia induction time. This may be because posterior lumbar plexus block anesthesia does not require sciatic nerve block, thereby reducing anesthesia risk, anesthesia time, and time to effect.

Posterior lumbar plexus block is difficult to obtain complete analgesic effect. Therefore, it is recommended to use it in combination with a sciatic nerve block, but combined use may lead to lower extremity muscle weakness and sciatic nerve damage. In this study, only posterior lumbar plexus block was used, and the perioperative hemodynamic indexes in this group were better than those in the control group. The results show that posterior lumbar plexus block anesthesia has advantages in maintaining perioperative hemodynamic stability in elderly patients with lower extremity fractures and helps to avoid abnormal fluctuations in blood pressure and heart rate. These results might be owing to the rapid absorption rate of anesthetics by the epidural space during epidural anesthesia, which easily leads to an excessive anesthesia plane and subsequent fluctuations in the circulatory and respiratory functions during the perioperative period, manifesting as abnormal changes in hemodynamic indicators. The posterior lumbar plexus block can avoid the above shortcomings [17]. Meanwhile, the lumbar plexus involves the obturator, femoral, and lateral femoral cutaneous nerves. Therefore, posterior lumbar plexus block anesthesia blocks all lumbar nerves and some sacral nerves. In addition, because the lumbar plexus block is located close to the spinal nerve, it can achieve the same effect as the spinal canal block [18, 19]. A posterior lumbar plexus block is only performed on one limb, which can reduce the hemodynamic fluctuations stemming from a sympathetic nerve block after intraspinal anesthesia and bilateral lower limb block [20, 21].

This study also explored the safety of posterior lumbar plexus block anesthesia in elderly patients with lower extremity fractures. The incidence of adverse reactions in the study group was slightly lower than that in the control group, indicating that posterior lumbar plexus block is safe. Therefore, posterior lumbar plexus block can allow patients to avoid prolonged hospitalization and increased treatment costs due to adverse reactions, which is essential for early recovery and discharge and lower hospitalization costs.

## 5. Conclusion

In summary, posterior lumbar plexus block anesthesia administered to elderly patients with lower limb fractures during surgical treatment maintained hemodynamic stability, shortened the block onset time and the anesthesia induction time, and reduced pain severity. However, we did not explore the effects of posterior lumbar plexus block anesthesia on the perioperative stress response from a microperspective using indicators, such as adrenaline and cortisol, which need to be further confirmed.

## Figures and Tables

**Table 1:** Hemodynamic index level comparisons between the study and control groups (mean ± standard deviation).

Projects	Groups	Cases	T_0_	T_1_	T_2_	T_3_
MAP (mmHg)	Study group	56	83.68 ± 7.25	89.33 ± 6.12	91.53 ± 7.29	88.09 ± 8.37
	Control group	56	85.01 ± 6.83	95.89 ± 7.17	96.65 ± 8.33	92.71 ± 7.51
	*T* value		0.999	5.208	3.461	3.074
	*P* value		0.320	0.001	0.001	0.003
HR (time/min)	Study group	56	80.20 ± 6.43	84.39 ± 7.51	83.67 ± 5.89	83.97 ± 6.15
	Control group	56	82.11 ± 7.91	88.62 ± 8.67	87.19 ± 6.77	86.72 ± 5.92	
	*T* value		1.402	2.760	2.935	2.411	
	*P* value		0.164	0.007	0.004	0.018	

**Table 2:** Anesthesia comparisons between the study and control groups (mean ± standard deviation).

Groups	Cases	BIS value			Onset time of retardation (min)	Anesthesia induction time (min)
		Anesthesia 5 min	Anesthesia 15 min	Anesthesia 30 min		
Study group	56	22.69 ± 6.91	28.19 ± 6.22	44.56 ± 5.96	3.17 ± 1.21	14.20 ± 2.93
Control group	56	30.29 ± 8.09	41.32 ± 9.01	53.45 ± 7.81	8.20 ± 2.87	23.38 ± 5.24
*T* value		5.346	8.974	6.772	12.085	11.443
*P* value		0.001	0.001	0.001	0.001	0.001

**Table 3:** VAS score comparisons between the study and control groups (mean ± standard deviation).

Groups	Cases	Preoperative	Immediately after surgery	6 h postsurgery	24 h postsurgery	48 h postsurgery
Study group	56	4.69 ± 1.23	3.48 ± 0.97	2.41 ± 0.89	2.01 ± 0.59	1.57 ± 0.49
Control group	56	5.01 ± 1.04	4.19 ± 1.00	3.10 ± 0.95	2.79 ± 0.70	1.99 ± 0.54
*T* value		1.487	3.814	3.967	6.376	4.310
*P* value		0.140	0.001	0.001	0.001	0.001

**Table 4:** The adverse reaction incidence rates of the study and control groups (*n* (%)).

Groups	Cases	Dizziness, headache	Low blood pressure	Vomiting, nausea	Respiratory depression	Skin rash	Total incidence
Study group	56	1 (1.79)	1 (1.79)	1 (1.79)	1 (1.79)	0 (0.00)	4 (7.14)
Control group	56	2 (3.57)	1 (1.79)	2 (3.57)	0 (0.00)	1 (1.79)	6 (10.71)
*χ* ^2^ value							0.439
*P* value							0.508

## Data Availability

All data was included in our manuscript.
